The article "Optimization of Human Motion Recognition Information Processing System Based on GA-BP Neural Network Algorithm" was retracted in 2023. Reasons: signs of a paper mill; suspected computer-generated content; unreliable results or conclusions; concerns about the data.

# Optimization of Human Motion Recognition Information Processing System Based on GA-BP Neural Network Algorithm

**DOI:** 10.1155/2021/1110503

**Published:** 2021-10-27

**Authors:** Shuwei Zhao

**Affiliations:** School of Physical Education, Xinxiang Medical University, Xinxiang, Henan 453003, China

## Abstract

At present, there are some problems in the process of human motion recognition, such as poor timeliness and low fault tolerance rate. How to effectively identify the motion process accurately has become a hot spot in the optimization system. In the existing research studies, the recognition accuracy is not very good and the response time is long. To end this issue, the paper proposed an information processing system and optimization method of human motion recognition based on the GA-BP neural network algorithm. Firstly, a human motion recognition system based on dynamic capture recognition technology is designed, which realizes the recognition of motion information from common postures such as action span, speed change, motion trajectory, and other aspects in the process of human motion. Secondly, the proposed algorithm is used to comprehensively analyse and evaluate the motion state. Finally, experiments are designed to verify and analyse the results. Compared to some baseline methods in human motion recognition information systems, the system in this paper based on the GA-BP neural network algorithm has the advantages of higher data accuracy and response speed, which can quickly and accurately identify the muscle group change in the process of human motion, and it can also provide customized motion suggestions based on the results.

## 1. Introduction

In recent years, the development of human motion recognition presents the trend of intelligence, modernization, and diversification [1]. For example, in basketball sports, many scholars have completed research on the athletes' movement state in the process of studying the athletes' bounce action and basketball shooting and mainly focused on action recognition and action prediction [2]. At present, the motion recognition methods provided by the existing motion training and motion recognition systems have certain limitations. It is difficult to select targeted sports training equipment according to their own muscle inertia and sports posture habits, so it is impossible to achieve the best effect of sports training and action optimization [3]. At the same time, the recognition accuracy is not very good and the response time is long.

To end this issue and find a good solution, this paper proposed an optimized information processing system of human motion state recognition. In the system, a GA-BP neural network algorithm is embedded. According to the difference in different movements of different groups of actions, posture and physical characteristics in the process of daily training and the detection and collection of the whole athlete's muscle group data through real-time body movement recognition and dynamic tracking can be collected and analysed.

In this paper, some contributions to human motion recognition have been made as follows:

1. A novel human motion recognition and dynamic tracking auxiliary training system based on the GA-BP neural network algorithm is proposed.
2. In this study, a human motion recognition system based on dynamic capture recognition technology is designed, which can realize the recognition of motion information from the common postures such as action span, speed change, motion trajectory, and other aspects in the process of human motion.
3. Compared to some baseline methods in human motion recognition, the designed system has the advantages of higher data accuracy and response speed, which can quickly and accurately identify the muscle group change in the process of human motion, and it can also provide customized motion suggestions based on the results.

The structure of this paper is presented as follows: In Section 1, the background is discussed and some motivations and contributions in this work are presented. In Section 2, some related papers in this field are described and their shortcomings have been pointed out. In Section 3, GA-BP neural network algorithm is constructed and applied to human motion recognition. In Section 4, some experimental results computed by the proposed model are discussed and analysed. In Section 5, some important achievements are concluded and the future work is included.

## 2. Related Work

In the past 30 years, there were many problems in research on human motion recognition information processing system, such as low efficiency, low recognition accuracy, and high error rate, especially in the construction of human motion recognition information processing system [4]. Gu et al. found that, in the process of strength training for most sports athletes, the recognition accuracy of the motion recognition system is not enough and it is unable to carry out large-scale training and feature recognition for specific muscle groups. Therefore, the research is carried out according to the game rules of sports and the theory of muscle training [5]. Abbas et al. first constructed a particle swarm optimization algorithm of the human motion state recognition system based on traditional sports training methods and adopted different weight allocation methods and recognition models to explain different athletes about the process of sports training. Based on kinematics theory and human movement recognition information management system, Zhou et al. proposed a hierarchical human movement state recognition method [7]. Through the research and analysis on the dynamic differences of weight, length, body fat, and strength of different athletes, Kim et al. proposed a new auxiliary recognition system of multimovement fusion based on principal component analysis [8]. To find out the difference between different human movement states and the influence of movement order on the overall sports training effect, Fadi et al. studied 800 sports lovers, simulated the “three-dimensional movement map” in the process of sports modeling drawing, and realized the basis of action evaluation in movement state recognition [9]. To solve the problems of low efficiency and effectiveness of motion recognition, Zhou et al. proposed a multiangle video recognition algorithm and a new athlete motion state recognition algorithm based on the fusion strategy technology of traditional sports training combined with Fourier function, so as to improve the recognition efficiency and stability of human motion [10]. To solve the problem of low efficiency in the process of human motion recognition, Li et al. proposed a semi-intelligent human motion recognition information analysis system based on neural network algorithm. However, the system is only applicable to the recognition of basketball and football, and not universal [11]. According to the fact that the accuracy of human motion recognition is interfered by light, Amaya et al. proposed a human motion recognition method based on infrared light, which can overcome the dependence on light intensity in the recognition process [12]. Zhao et al. found that some actions in the process of human movement have certain similarities; hence, a motion capture recognition model for specific actions is proposed, which can recognize a certain kind of specific motion with high accuracy [13]. According to the differences in the human body, Zhang et al. proposed a customized human motion recognition information system, which can effectively adjust dynamically according to the differences of human height, so as to improve the recognition efficiency and accuracy, but the use of the system is greatly affected by the motion scene [14]. According to the differences of human movement types, Geist et al. proposed a human movement recognition model for the elderly, which can effectively identify the movement posture and stability of the elderly and can play a certain early warning function for the physical quality of the elderly [15]. To sum up, it can be seen that most of the current human motion state recognition models do not involve the construction of the GA-BP neural network algorithm and sports auxiliary training system based on motion state dynamic capture and training data. There are relatively few research results on the precise recognition, specific quantitative training dynamic evaluation system, and action in the process of motion state recognition [16]. Moreover, there is no construction of the motion recognition information processing system for specific groups or specific movements [17].

In the mentioned papers, most of them did not try to use an artificial intelligence (AI)- powered algorithm to study the human motion recognition, especially in sports fields. Of course, some scholars used the AI model, but the recognition accuracy is not very good and the response time is long.

## 3. Optimization of the Human Motion Recognition Information Processing System Based on GA-BP Neural Network Algorithm

### 3.1. Application of GA-BP Neural Network Algorithm in the Human Motion Recognition Information Processing System

Up to now, neural network algorithms have been optimized in different dimensions and have been applied in many fields. In this paper, the GA-BP neural network algorithm as an intelligent algorithm is applied to the optimal path in the process of human motion state recognition [18, 19]. In order to more intelligently and accurately analyse the influence of human movement state on recognition accuracy, this study refers to the optimization strategy of neural network application in other fields and adopts the optimized GA-BP neural network algorithm to recognize and analyse the body movement characteristics of athletes in the process of movement [20]. In addition, research studies have shown that the distortion measure of the GA-BP neural network algorithm can be compensated [21]. The reference indexes of common neural network algorithms are shown in Table 1.

Combined with the above idea of GA-BP neural network, in this study, in the aspect of human action recognition, using the local search and classification algorithm based on GA-BP neural network factors, three characteristic parameters related to the identification of physical characteristics and movement state of sports athletes are selected. A motion recognition information processing system based on the recognition characteristics of athletes' body movements is constructed. Through the research of daily motion decomposition, motion analysis, and motion trajectory capture, we explore the establishment of intelligent human motion recognition information processing system from multiple perspectives and then classify and analyse the characteristics of athletes' multiple motion recognition results by combining the GA-BP neural network algorithm.

### 3.2. Human Motion Recognition Process Based on GA-BP Neural Network Algorithm

In order to realize the construction of human motion recognition information processing system, it needs to be divided into three steps: human motion recognition, recognition information extraction, and information data standardization. In the process of human motion recognition, the decomposition and efficient processing of the action to be recognized can be realized according to the hierarchical difference pattern. In the step-by-step solving process, it can be distinguished by identifying the value of the precision function and the expression *y*(*x*) is

(1) $$\begin{array}{c} y\left(x\right)=\frac{y\left(x-1\right)x^{2}}{n_{R}+1}\left(x+1\right), \end{array}$$

where *x* is the action data and *n*_*R*_ is the reference value of the human body. In this process, we need to complete the calculation of *y*_*n*+1_. In fact, we have worked out a series of approximate values *y*_0_, *y*_1_,…, *y*_*n*_. If we make full use of the information of human movement differences to predict *y*_*n*+1_, we can expect to obtain higher accuracy. Therefore, if the initial value is known, the eigenfunction can be solved according to the linear chain method:

(2) $$\begin{array}{c} t\left(x_{i}\right)=h\sum_{i=1}^{n}\frac{y{\left(x_{n+i}\right)}^{2}}{y\left(x_{n+i-1}\right)+y\left(x_{n+i+1}\right)}, \end{array}$$

where *h* is the conventional coefficient. When we randomly process a single neuron structure with multiple neuron structures (nodes) (in this paper, we refer to highly correlated human movement), the processing process will be as shown in Figure 1.

After the completion of the above links, the mutual coupling analysis of the two-way sports training morphological structure and the vector processing analysis of multiple coupling combinations are carried out to achieve accurate identification and analysis of the overall movement state and then multiple structural morphological features with high similarity of movement structure are found from the total sports athletes group [22]. After many rounds of comparative analysis, the new generation of people with the characteristics of overlapping movement morphology growth needs movement morphology structure. A specific human motion state model that meets the recognition conditions is finally generated; that is, the analysis value of the normal boundary of a certain motion state is close to the normal demand value of the actual motion state. In this way, the unique motion state can be captured under the condition of the GA-BP neural network algorithm and the integrated shape recognition in the training process can be realized [23]. The reference indexes of the integrated morphological recognition analysis are shown in Table 2.

### 3.3. Construction Process of the Human Motion Recognition Information System Based on GA-BP Neural Network Algorithm

Because the human motion recognition information system needs to realize the capture, detection, and intelligent analysis of sports athletes' motion state (that is, the basic function of the system), we use the step model based on the fork tree structure to realize this process. In this process [24], GA-BP neural network realizes process characteristics of different human movement processes, which is based on a large number of human movement shape characteristics (such as normal juvenile movement shape, youth movement shape, male movement shape, and female movement shape) [25]. Then, we get the values of motion capture, detection, and analysis in this category and classify the optimal training morphological data objects that meet the standard value. The classification function *r*(*x*) is

(3) $$\begin{array}{c} r\left(x\right)=d_{2}*\;\cos\left(\frac{90*\left(x-2\right)}{x+2}-\frac{180}{d_{2}x}+\frac{360}{x}\right), \end{array}$$

where *x* is the action data and *d*_2_ is the threshold reference value. Therefore, aiming at the motion state capture, dynamic motion analysis model, and sports auxiliary training system, we will first use the existing normal motion form big data information and intelligent analysis and processing [26]. The specific value range of the initial weight and the lowest threshold reference value of the motion recognition form requirement degree needed in the GA-BP neural network algorithm is obtained. Then, the GA-BP neural network algorithm is used to decompose different sports actions in three dimensions, and the decomposition function *e*(*x*) is

(4) $$\begin{array}{c} e\left(x\right)=\frac{g*m_{1}*m_{2}}{x^{2}}, \end{array}$$

where *x* is the action data, *m* is the reference value of different dimensions, and *g* is a nonzero fixed constant. Next, it is necessary to complete the recognition and intelligent analysis of the demand degree of the standard action form with secondary subdivision, finally obtain the optimal solution search, and then screen out the best recognition form and sports action capture screening range. The process is shown in Figure 2.

Based on this, the disturbance degree of the identification process is judged firstly, and if the disturbance degree is within the controllable range, the method is said to be stable and the disturbance correction function *l*(*x*) for detecting the disturbance degree is

(5) $$\begin{array}{c} l\left(x\right)=\sqrt{\frac{3x^{3}+4x^{2}+7x+2}{4x^{3}+3x^{2}+8x+1}},\\ l\left(x\right)=y\left(x\right)e^{\lambda \left(x-3\right)}. \end{array}$$

Among them, *λ* is the disturbance reference value. After completing the above steps, combined with the current human age database and the posture database of common movements, the initial self-test of the recognition process of human movements in this system is carried out. The simulation process and results are shown in Figure 3. From the simulation results, it can be seen that the recognition process of human movements has a high degree of coincidence.

The motion state capture technology model in the human motion recognition information processing system can display the difference of the detected person's motion shape in sports and after sports, unify the difference of the human carpal bone shape in different sports with the time length of the motion recognition link, and carry out different degrees of weight analysis and processing [27, 28].

As can be seen from Figure 3, all models have the same change trend and the peaks and troughs appear at exactly the same point because all three models are computed in the same samples and the proposed model includes some features of the other two baseline methods. Overall, compared to the other two baseline methods, the recognition results of the human motion recognition system based on the GA-BP neural network have a good stability and reliability. It can be seen that the error of state structure stability network processing result of motion recognition is significantly reduced.

### 3.4. Optimization Process of the Human Motion Recognition Information System

After the construction of human motion recognition information system, in order to further improve the recognition efficiency and accuracy, we need to further optimize the human motion recognition information process. First of all, according to the theory of motor neurology, we can learn from a new model to analyse and self-study the cooperation degree of sports state relationship in the process of traditional sports. The analysis process is shown in Figure 4.

Secondly, according to different types of human motion rules and action recognition efficiency, multidimensional decomposition of different types of human motion models can be realized, which can produce auxiliary and reference functions for the human motion recognition system in the process of recognition, which indicates that the actual fitness of the human movement shape analysis model is very high, that is, the more reliable the recognition and analysis record of the movement state of an individual in the process of sports. The simulation results are shown in Figure 5. The simulation results show that the data stability is improved significantly and data can be stabilized at the set threshold of “1”.

Finally, it is necessary to control the error of the identified motion state. This process uses the commonly used error analysis function *h*(*x*), whose expression is

(6) $$\begin{array}{c} h\left(x\right)=\frac{\sum_{i=1}^{n}{\left(x_{i}-\bar{x}\right)}^{2}}{n\bar{x}}. \end{array}$$

Among them, *x* is the action data of recognition. The reference standard of secondary identification verification mechanism is shown in Table 3.

## 4. Experimental Results and Discussion

### 4.1. Experimental Verification of the Human Motion Recognition Information Processing System Based on GA-BP Neural Network Algorithm

In order to verify the optimization performance, it is necessary to set up relevant experiments. Considering the differences between the experimental samples and the actual movement situation, this study uses a sufficient number of random experimental samples and carries out at least 120 repeated experiments, so as to eliminate the impact of random errors and increase the credibility of verification experiments. Under the information processing system of sports state recognition, different ways of sports forms correspond to different sports states, such as the differences of athletes, sports differences of different age stages, sports forms of different genders, and sports differences of different regions. The experimental results are shown in Figure 6.

Whether the action form of the tested person meets the corresponding form of standard sports action is mainly based on the automatic comparison and analysis of normal action forms at the big data level. Firstly, the system and automatic two-way information are compared with each other, and then the detection and accurate processing of key motion attitude feature data are realized. That is to say, if the corresponding weights are different, the greater the correlation is, the greater the corresponding weights will be, so as to realize the analysis of specific sports and the identification of sports forms. This intelligent comprehensive evaluative verification experiment based on big data analysis does not need to label and screen specific groups in advance but only needs the motion state recognition system based on the GA-BP neural network algorithm to complete the experimental process.

In the process of experiment, we need to optimize the motion morphology analysis model based on multiple comparative analysis and screening, first receive the external similar features of the same kind of motion morphology structure, then carry out data processing to obtain the relevant unique vector group, and finally obtain the evaluation sample data of different motion recognition processes. The optimized GA-BP neural network algorithm needs the initialization weight and the lowest prediction threshold of normal motion structured data. The preliminary test data of specific experimental samples are shown in Figure 7.

From the experimental results in Figures 6 and 7, it can be seen that the optimized human motion recognition information processing system (GA-BP) has better overall effect and higher recognition accuracy. Compared to the other two baseline methods (GA and BP neural network), the proposed model also has better data stability and recognition speed. This is because GA-BP neural network algorithm will not progress in the local optimal value in the search iteration process, and in the process of optimizing the initialization weight and the actual threshold of GA-BP neural network algorithm, the optimal vector obtained is inversely transformed and the data processing efficiency is faster. In all three models, the BP neural network shows the worst performance in the recognition accuracy, but its recognition speed shown in Figure 7 is better than the GA model, because the GA model will progress in the local optimal value in the search iteration process more easily.

### 4.2. Analysis of the Experimental Results of the Optimized Motion State Recognition Information Processing System

In this paper, the test object is the action form of the standard sports action randomly selected from the multigroup movement state form of the same age, the same gender, and the same area. The data consistency of the test and analysis results is shown in Figure 8. It can be seen from Figure 8 that the stability of the proposed model and BP neural network is better than that of the GA model. In all three models, the proposed model has the smallest errors.

The initial value analysis is used for the experimental process, and the analytical solution of the initial value problem is *y*(*x*)=*e*^−15*x*^; then, we use the third order, fourth order, fifth order, and sixth order to solve the relevant results of the experimental object in this model. The numerical results of error in different levels are shown in Table 4.

The experimental results show that the third-order, fourth-order, and fifth-order neural network algorithms constructed in this paper are feasible. The solution stability (dimensionless index) of the experimental results of sports state structure recognition is shown in Figure 9.

As can be seen from Figure 9, the experimental results show that compared to the experimental stability, the system (GA-BP) can more effectively reduce the error of action search matching block in the process of motion recognition; therefore, it effectively improves the recognition efficiency and recognition accuracy.

## 5. Conclusion

The traditional human motion recognition information processing system has the problems of low recognition efficiency, poor stability, and poor reliability, and the intelligent model is based on iterative analysis algorithms. They also have low utilization of digital information and digital conversion rate. Therefore, the traditional human body motion state recognition method can no longer meet the current human motion recognition information processing requirements. To end this issue, this paper proposed the information processing system and optimization strategy of human motion recognition based on the GA-BP neural network algorithm. This paper first discussed the status and problems of sports action recognition and then designed a motion state recognition and training model based on motion capture technology and the GA-BP neural network algorithm. According to the different influence degrees of the model on the recognition process, the comparative experiments show that the error of the motion information processing system identified by this model is within the stable standard reference range, and compared to other baseline methods, its recognition accuracy and recognition speed are significantly improved. The experimental results show that the model can judge whether there is a problem of nonstandard movement of athletes with similar characteristics through the results of movement state recognition. However, this model only considers the effect of action recognition and does not consider the influence of other factors; so, there is a room for improvement in the future.

## Figures and Tables

**Figure 1:** Data processing process of the neural network model.

**Figure 2:** Screening out the best movement recognition morphology process.

**Figure 3:** Initial self-check simulation process of the human body motion recognition data.

**Figure 4:** Analysis process of the degree of cooperation of the motion state relationship.

**Figure 5:** Data stability of simulation results. (a) Simulation group (b) Simulation control group.

**Figure 6:** Experimental simulation analysis results.

**Figure 7:** Experimental test data image output.

**Figure 8:** Action recognition stability results of experimental data.

**Figure 9:** Action recognition stability results of experimental data.

**Table 1:** Common reference indicators for neural network algorithms.

Reference indicator	Neural networks	BP neural networks	GA-BP neural networks
Number of neuron nodes	>3	>10	>15
Number of hidden layers	>4	>6	>8
Number of cross validations	>5	>7	>9

**Table 2:** Reference index for holistic pattern recognition and analysis.

Reference indicator	GA-BP neural networks (%)	Absolute error
Movement speed	87	0.005
Sports profile	85	0.005
Action feature extraction	90	0.005

**Table 3:** Reference standard for secondary identification verification mechanism.

Reference indicator	Initial verification	Secondary verification
Difference between recognition result and threshold	0.1	0.05
Difference between recognition speed and threshold	0.2	0.05

**Table 4:** Experimental data results.

Method	3rd-order solution	4th-order solution	5th-order solution	6th-order solution
GA-BP neural networks	3.588*E* − 033	2.941*E* − 033	2.6282*E* − 033	0.8102*E* − 002
GA neural networks	3.951 − 033	3.7086*E* − 033	3.1954*E* − 033	1.1285*E* − 002
BP neural networks	3.842*E* − 033	3.6868*E* − 033	3.1563*E* − 033	1.1312*E* − 002

## Data Availability

The data used to support the findings of this study are available from the corresponding author upon request.
